The article "Tracheal Bronchus: A Rare Etiology of Recurrent Pneumonia in Children" was retracted in 2024. Reasons: false authorship; unreliable results or conclusions; no approval from an author; concerns about the authorship.

# Tracheal Bronchus: A Rare Etiology of Recurrent Pneumonia in Children

**DOI:** 10.7759/cureus.20378

**Published:** 2021-12-13

**Authors:** Saif A Alqahtani, Anwar M Alghamdi, Rawan A Babader, Doaa A Aljehani, Razan K Alsultan, Rawiah Y Mushari, Maha Y Alyahya, Hawra I Alajwad, Ahmad A Alibrahim, Egbal B Altukruni, Reem N Alhasani, Arwa T Mandurah, Yara A Halabi, Batool J Alghamdi, Faisal Al-Hawaj

**Affiliations:** 1 College of Medicine, Jordan University of Science and Technology, Irbid, JOR; 2 College of Medicine, Ibn Sina National College for Medical Studies, Jeddah, SAU; 3 College of Medicine, AlMaarefa University, Ad Diriyah, SAU; 4 College of Medicine, Jazan University, Jazan, SAU; 5 College of Medicine, King Saud University, Riyadh, SAU; 6 College of Medicine, Arabian Gulf University, Manama, BHR; 7 College of Medicine, Medical University of Warsaw, Warsaw, POL; 8 College of Medicine, Qassim University, Qassim, SAU; 9 College of Medicine, Umm Al-Qura University, Mecca, SAU; 10 College of Medicine, Imam Abdulrahman Bin Faisal University, Dammam, SAU

**Keywords:** case report, computed tomography, recurrent pneumonia, rare congenital anomaly, tracheal bronchus

## Abstract

Recurrent infections are a common cause for seeking medical care and they result in significant parental anxiety and concerns. Although immunodeficiency disorders are an important underlying cause of recurrent infections, the majority of children with recurrent infections do not have any dysfunction in their immune systems. We present the case of an 11-year-old boy who was brought to the outpatient department by his parents because of a complaint of productive cough for the last one week that was associated with low-grade fever. The patient had a history of frequent episodes of pneumonia. He developed three episodes of pneumonia within the last year. According to the parents, the patient was investigated previously for possible immunodeficiency disorders, but the findings did not reveal any abnormal results. His siblings are healthy and have no history of recurrent infections or immunodeficiency disorders. The vital signs were within the normal limits. The patient was treated empirically with the antibiotic course of amoxicillin. The patient was given a follow-up appointment one week later. In the follow-up visit, the patient had complete resolution of the infection. The parents expressed concern about their child having recurrent episodes of infections. The patient underwent a high-resolution CT scan of the thorax to rule out any structural abnormalities. The scan demonstrated the presence of an aberrant bronchus arising from the lateral wall of the trachea above the level of the carina and supplying the apical segment of the right upper lobe. This finding is often referred to as a “tracheal bronchus.” The tracheal bronchus is a rare congenital anomaly of the respiratory tract. It should be considered in the differential diagnosis of children with recurrent pneumonia with no infections in other organ systems to suggest immunodeficiency disorder.

The article "Tracheal Bronchus: A Rare Etiology of Recurrent Pneumonia in Children" was retracted in 2024. Reasons: false authorship; unreliable results or conclusions; no approval from an author; concerns about the authorship.

## Introduction

The history of recurrent infections in a child can be associated with significant parental concern. Recurrent infections are defined as having three or more respiratory infections in one year or having two or more severe infections in one year [1]. While immunodeficiency disorders are an important cause of recurrent and severe infections, the majority of children with recurrent infections do not have any dysfunctions in the immune system. Further, a prior study showed that only 10% of children with recurrent infections have immunodeficiency disorders [2]. Additionally, up to 50% of children with recurrent infections are not found to have any condition explaining their infections [1]. It is essential to note that the majority of patients with recurrent infections who are localized to a single organ system usually have structural abnormalities or chronic diseases, rather than an immunodeficiency disorder. Patients with recurrent pneumonia should be carefully evaluated based on the pattern of their infections. For example, children with recurrent pneumonia in different lung regions are most likely to have immunodeficiency disorders. In contrast, children with recurrent pneumonia in a similar location typically have anatomic abnormalities such as foreign bodies [3]. Here, we present the case of an 11-year-old boy with recurrent pneumonia that was diagnosed as having a tracheal bronchus, a rare congenital anomaly of the respiratory system.

## Case presentation

We present the case of an 11-year-old boy who was brought to the outpatient department by his parents because of a complaint of cough for the last one week. His cough was productive of yellowish sputum, but it did not contain any blood. The cough was associated with fever that measured 38.1℃ and was not improved by over-the-counter analgesics. There was no history of chest pain, shortness of breath, or wheezing.

The patient had a history of frequent episodes of pneumonia. He developed three episodes of pneumonia within the last year. According to the parents, the patient was investigated previously for possible immunodeficiency disorders, but the findings did not reveal any abnormalities. There was no history of recurrent infections other than pneumonia. No history of recurrent otitis media, gastroenteritis, or skin infections. He did not undergo any previous surgeries. His growth and developmental history were unremarkable for any concern. He was up-to-date with the vaccination schedule. The antenatal history of the patient was non-contributory. The patient was not born of consanguineous marriage. His siblings are healthy and have no history of recurrent infections or immunodeficiency disorders. The family history was remarkable for asthma.

The article "Tracheal Bronchus: A Rare Etiology of Recurrent Pneumonia in Children" was retracted in 2024. Reasons: false authorship; unreliable results or conclusions; no approval from an author; concerns about the authorship.

Upon examination, the child was well nourished and there were no signs of respiratory distress. The vital signs were within the normal limits. He had a pulse rate of 100 beats per minute, respiratory rate of 21 breaths per minute, temperature of 37.0℃, and blood pressure of 100/65 mmHg. His oxygen saturation was normal. Chest examination revealed normal air entry bilaterally with scattered crepitations. Basic laboratory investigations were performed and showed no abnormalities (Table 1). Chest X-ray revealed airspace opacity in the right upper lobe (Figure 1). Hence, the patient was treated empirically with the antibiotic course of amoxicillin. The patient was given a follow-up appointment one week later.

**Table 1:** Summary of the results of laboratory findings.

Laboratory investigation	Unit	Result	Reference range
Hemoglobin	g/dL	14.5	13.0–18.0
White blood cell	1000/mL	4.5	4.0–11.0
Platelet	1000/mL	388	140–450
Erythrocyte sedimentation rate	mm/hr.	3	0–20
C-Reactive Protein	mg/dL	2.4	0.3–10.0
Total bilirubin	mg/dL	0.4	0.2–1.2
Albumin	g/dL	3.9	3.4–5.0
Alkaline phosphatase	U/L	50	46–116
Gamma-glutamyltransferase	U/L	17	15–85
Alanine transferase	U/L	16	14–63
Aspartate transferase	U/L	15	15–37
Blood urea nitrogen	mg/dL	9	7–18
Creatinine	mg/dL	0.9	0.7–1.3
Sodium	mEq/L	137	136–145
Potassium	mEq/L	3.8	3.5–5.1
Chloride	mEq/L	106	98–107

**Figure 1:** Chest radiograph demonstrates airspace opacity (long arrow) in the right upper zone. Also, a radiolucency branching of the trachea is noted (small arrow) that is suggestive of a tracheal bronchus. Note: the possible finding of tracheal bronchus in this image was not recognized by the treating physicians before the CT scan.

In the follow-up visit, the patient had complete resolution of the infection. The parents expressed concern about their child having recurrent episodes of infections. Despite their several visits to different clinics, no explanation for the recurrent pneumonia was given. In order to rule out any structural abnormalities or the possibility of a foreign body, the patient underwent a high-resolution CT scan of the thorax. The scan demonstrated the presence of an aberrant bronchus arising from the lateral wall of the trachea above the level of the carina and supplying the apical segment of the right upper lobe. This finding is often referred to as a “tracheal bronchus” (Figures 2-3).

The article "Tracheal Bronchus: A Rare Etiology of Recurrent Pneumonia in Children" was retracted in 2024. Reasons: false authorship; unreliable results or conclusions; no approval from an author; concerns about the authorship.

**Figure 2:** Axial CT image demonstrates the aberrant bronchus (arrow) originating from the trachea.

**Figure 3:** Coronal CT image demonstrates the aberrant bronchus of the apical segment of the upper lobe (arrow) originating directly from the trachea.

The radiological findings were discussed with the parents. The available management options were given. The option of surgical intervention with segmentectomy or lobectomy was discussed. However, the parents refused any surgical intervention.

## Discussion

We presented the case of a young child with recurrent pneumonia due to tracheal bronchus, which is a rare congenital anomaly of the respiratory tract. The tracheal bronchus refers to a group of anatomic variations in which the upper lobe had a bronchus originating directly from the trachea. The origin of such bronchus may be from the cricoid cartilage to the carina [4].

The exact explanation of the development of tracheal bronchus is incompletely understood. It is suggested that the tracheal bronchus arises from a migration of a part of a previously developed bronchus to a different site on the trachea. A previous study suggested that the prevalence of such anomalies is less than 1% among children [5].

Several congenital anomalies have been described in patients with a tracheal bronchus. Such associations included Down syndrome, esophageal atresia, neural tube defects, congenital heart disease, VATER association, and hypoplastic lung [5-6]. In the present case, however, the patient did not have any history of congenital anomalies, and his past medical history was unremarkable apart from the history of recurrent pneumonia.

The site of pneumonia is crucial to define the diagnostic pathway among children with recurrent pneumonia. In the present case, the parents reported that they had several previous visits for recurrent pneumonia and extensive investigations to exclude any primary immunodeficiency disorders. However, the patient should have been investigated for the presence of anatomic anomalies as he had no history of infections in other organ systems [7]. As in our case, a CT scan of the chest with multiplanar reconstructions in the coronal plane allows making the diagnosis easily.

The aberrant course of the tracheal bronchus makes it vulnerable to obstruction. This can result in lobar collapse and infection. Hence, it is unsurprising to encounter patients with tracheal bronchus to present with recurrent pneumonia as in our case [7]. Previous research showed that some patients with tracheal bronchus present with wheezing because of the narrowed aberrant bronchus and is often misdiagnosed as asthma. Few cases reported showed an association of tracheal bronchus with pulmonary tuberculosis and malignancies [4].

The article "Tracheal Bronchus: A Rare Etiology of Recurrent Pneumonia in Children" was retracted in 2024. Reasons: false authorship; unreliable results or conclusions; no approval from an author; concerns about the authorship.

## Conclusions

The tracheal bronchus is a rare congenital anomaly of the respiratory tract. It should be considered in the differential diagnosis of children with recurrent pneumonia with no infections in other organ systems to suggest immunodeficiency disorder. Appropriate investigation for tracheal bronchus is warranted in pediatric patients with recurrent infection localized to the same region.
